# Cloud Computing Load Balancing Mechanism Taking into Account Load Balancing Ant Colony Optimization Algorithm

**DOI:** 10.1155/2022/3120883

**Published:** 2022-04-12

**Authors:** Jing He

**Affiliations:** College of Artificial Intelligence and Big Data, Chongqing Industry Polytechnic College, Chongqing, China

## Abstract

The networking scale and traffic have exploded. At the same time, the rapid development of virtualization and cloud computing technologies not only poses a considerable challenge to the endurance of the network, but also causes more and more problems to the traditional network architecture with IP as the core. Cloud computing is a supercomputing model based on the Internet. With the rapid growth of network access and data traffic, the processing power and computing intensity will also increase, and a single server cannot afford the increase in business. In order to reduce network pressure and improve computing efficiency, load balancing for network computing is particularly important. This paper uses ant colony algorithm to design cloud computing load balance. The ant colony algorithm runs in the controller. According to the real-time network load situation provided by the controller, it calculates the link with the smallest load and provides a dynamic data stream forwarding strategy. The result of the experiments shows that the load-balanced ACO optimized technique can significantly provide an improved computational response. In the ACO algorithm, the average response time is about 30% lower than that in other algorithms. This shows that the use of the ant colony algorithm achieves a good optimization effect.

## 1. Introduction

Cloud computing is a relatively new technology based on software services such as electricity and computing. It does its job by providing service and feedback. Service provision and use conditions are important features that distinguish it from the previous complex. Low database efficiency will affect system performance, reduce system response time, and even more seriously cause node downtime. For the scheduling of cloud resources, the diversity of cloud components and the diversity of user needs make some nodes overloaded, affecting the use of the entire system and resources. Cloud computing can realize the sharing of resources, can process massive amounts of data, and can provide an unlimited amount of storage space. Therefore, cloud computing is applied to military, school, medicine, scientific research, and other fields. However, when cloud computing faces such a large number of users, it has to deal with a lot of data and tasks. When a large number of requests are processed at the same time, this will affect the performance of the entire system. Therefore, how to achieve source access load balancing has become one of the most important issues in the implementation of cloud computing.

Cloud computing is already a significant area of research as a computer scientist. Load balancing technology is considered to be one of the most vital research directions in cloud computing and is a popular research direction that is constantly evolving. In cloud computing, the evolution must rely on the development of load balancing technology. So far, there is no ideal research result for downloading load balancing technology used in cloud environment, so it can be studied from different aspects. Due to its positive feedback mechanism and robustness, ant colony algorithm has been extensively studied and improved since it was proposed, especially for combinatorial optimization problems in application. Ant colony algorithm shows great advantages, so this article will use ant colony algorithm as the basis to apply it to the resource allocation problem in cloud computing.

A large amount of research has been done by domestic and international experts on the application of ant colony algorithms. Zhao et al. proposed a fault classification technique for neutral and invalid grounding systems based on binary ant colony algorithm (BACA) with fuzzy neural network (FNN). Test samples and field experimental findings indicate the high accuracy and good adaptability of the proposed fault classification method [1]. Vu et al. proposed the development of a quantum ant colony algorithm (QACA) to improve silent human transmission from dangerous areas to safe areas. Compared to the ACO (ant colony optimization) method, QACA has the ability to find better solutions faster using fewer individuals due to quantum representation and pheromone information and has a stronger potential. Experimental results show that the proposed method has more effective performance [2]. Pham et al. proposed a new algorithm that combines scene filtering procedures, precise algorithms, and parallel ant colony algorithms. Experiments show that building multiple initial solutions with reduced scene sets for the ant colony algorithm can significantly reduce the total time required to find the best solution. The proposed algorithm can be used for the automated construction of reliable control systems [3]. Jiang et al. used the ACO algorithm, which uses anaerobic digestion (AnD) for combination to increase biogas production to increase the release of organic waste from various waste sources in real time. An enrichment plant has been developed based on a virtual case study of organic waste affecting urban wastewater treatment plants and agri-food operations. Studies have shown the importance of the ACO method in supporting decision-making processes that help improve organic waste management and SWS control [4]. As for load balancing methods, there are fewer related studies. Hajiesmaili et al. proposed a traffic load balancing framework that seeks to strike a balance between network applications (such as total delivery delays) and green energy consumption. The statistical results show that the proposed traffic load balancing process can achieve adjustable compensations between the use of grid power and the total traffic delivery delay and saves a lot of network-connected energy at a certain cost [5]. Sarma et al. reviewed the program documentation proposed by current load balancing technologies. In addition, the advantages and disadvantages associated with many load balancing algorithms are also discussed, and the main challenges of these algorithms are identified, so that more efficient load balancing systems can be developed over time [6]. Akbari et al. proposed another algorithm with less complexity for the load balancing problem. The algorithm provides worst-case performance guarantees and describes a simple way to approximate user associations for a given input by a bias factor. Next, there is a small-scale algorithm for the overall optimization problem, with an algorithm based on the following approximate method, which has been used for nonextension optimization problems [7]. Zhao J proposed a new heuristic method for the physical host selection problem of the deployment request task, which is called Bayesian and clustering-based load balancing. As demonstrated by the results of the simulation, the proposed approach significantly reduces the failures of the mission deployment incidents, improves the amount of throughput, and optimizes the outside-in service performance of the hybrid service in the cloud data center compared to existing work [8]. These studies provide a great reference for this article, but there are few studies on the application of ant colony optimization algorithms to cloud computing loads.

The article introduces the basic knowledge of cloud computing and the problem of resource allocation in the cloud computing environment. The objective function is proposed, and the improved genetic ant colony algorithm proposed is applied to the resource allocation problem. The operation steps and process of the algorithm are listed in detail. We integrate file size, file access speed, CPU performance, memory size, bandwidth, and other factors and perform data migration based on comprehensive load. The article takes the functional characteristics of the cloud computing platform as the background and, on the basis of the preliminary development of the current cloud computing platform resource management technology, further researches the elastic load balancing technology under the cloud computing platform.

## 2. Cloud Computing Load Balancing Method

### 2.1. Cloud Computing

Cloud computing is a supercomputing model based on the Internet. It realizes the sharing of resources, and the resources and software in the cluster are allocated to users on demand. The goal of cloud computing is based on network technology to bring together traditional scattered computers to form a cluster. This combined cluster strengthens the processing capacity of the entire system.

The basic idea of cloud computing is that, in a distributed computing environment, each user can freely find the services he/she needs in this system quickly [9]. How to improve the average service response rate of the system has become a crucial issue in cloud computing [10]. The results of the cloud computing system are shown in Figure 1.

Cloud computing can be roughly divided into three categories, called the SPI model: software as a function, platform as a function, and infrastructure as a function. The infrastructure as a service provides the basis for platform services [11]. The platform as a service uses the infrastructure as a service to provide software as a service [12]. The platform as a service is similar to the web hosting service in the web hosting market. The corresponding relationship is shown in Figure 2.

Cloud computing has the following three characteristics:

1. Cloud computing is based on virtualization technology to realize rapid deployment of resources and access to services.
2. Cloud computing is provided to users in the form of services that are oriented to massive amounts of information and provided through the Internet.
3. The resources of cloud computing can be dynamically expanded and configured according to the needs of users and paid according to the actual use of users. Users do not need to manage them themselves, which can reduce the burden of users' processing and dependence on IT expertise.

Cloud storage uses grid technology, aggregation technology, or file sharing technology to fully organize and coordinate multiple clouds of different storage devices on each device in the cloud-covered data center [13]. Cloud storage is a cloud computing storage system. User data is stored in the cloud. For users, local storage systems and storage devices are not required [14]. More specifically, cloud storage is a service in which data is provided by a collection of multiple storage devices and servers, and users purchase services on demand.

Cloud storage deals with massive amounts of data, and it is necessary to complete the storage and management of massive amounts of data. The storage layer is composed of storage devices and storage device management systems. The storage application management system mainly completes the maintenance and upgrading of storage facilities and the monitoring of storage equipment. The structure of the cloud storage system is shown in Figure 3.

Cloud data centers usually include thousands of servers; these server nodes are heterogeneous and unevenly distributed. The storage and scheduling of resources are coordinated by many servers, and the user's access to the server is random, diversified, and complicated. The existence of these factors can easily cause some server nodes to be idle. While other server nodes are in a state of overload saturation; that is, the load of server nodes is not balanced. The load of server nodes includes not only the load of data storage, but also the load of resource scheduling. Obviously, the existence of this imbalance will cause a waste of cloud resources, increase the burden on the network, and affect the use of users. Therefore, it is essential that the issue of load balance in relation to cloud computing is addressed. A suitable load balancing strategy allows for optimal configuration of services and increased working power.

### 2.2. Load Balancing Algorithm

Load balancing is realized by monitoring the usage of resources on each physical node and then analyzing the collected resources; by analyzing the algorithm of load balancing, the load on the node is dynamically migrated to the node with a small load; and finally the purpose of load balancing is achieved. Any computer or server source can be optimized, the response time can be as short as possible, and the processor performance can be as high as possible. Under normal circumstances, the user partition is finally obtained by analyzing the source of each controller (such as CPU usage, memory space, and bandwidth). Normally, the architecture of load balancing is shown in Figure 4.

A load balancing system is mainly composed of three parts: the cloud platform of the IaaS layer realizes the collection of resources, the realization of the load balancing strategy in the PaaS layer, and the web customer service terminal of the SaaS layer makes requests. At the IaaS layer, the underlying virtualization is mainly realized through the OpenStack cloud platform, and the monitoring function is mainly used to monitor and collect the resources of each node through Ganglia.

The PaaS layer is the core module to achieve load balancing, which is achieved through load balancing based on the dynamic load balancing algorithm mentioned in Section 3. In this layer, the dynamic scheduling of virtual machines on the nodes is realized through WSO2 software. The PaaS layer is mainly used to implement load balancing strategies and scheduling. The core processing module is the strategy controller and the queue manager. The strategy selection is mainly to analyze the load data collected by the server. By analyzing which physical machines and virtual machine resources are overloaded, underloaded, etc. and saving the data in the database, the corresponding data needs to be fetched from this database during scheduling. However, the queue manager mainly queues data.

Common load balancing algorithms include round-robin balancing algorithms, weighted round-robin symmetry, temporary balancing algorithms, and mechanical balancing algorithms.

The rotation balance algorithm used is to determine the rotation frequency before sending the request and then divide the request, rotation, etc. on the respective servers according to this process.

At the weighted round-robin balancing algorithm, the performance of each server is not considered in the round-robin balancing algorithm. The performance of each server is inconsistent, and greater configuration and processing capacity mean greater weight; then, the load allocated to the server will be more, and the higher the load, the more efficient the operation.

The concept of load balancing is first introduced at each server node in the static payload trading algorithm, and then the corresponding function is allocated to each server, rather than the estimated resource power allocation. In the process of adjusting the concept and load balancing, the load status of each server is taken, but a value is assigned to the load, and this value will not change with the change of the load.

Consequently, the dynamic burden balancing method is a very good solution. The animated workload trading algorithm overcomes the weaknesses of static payload trading. The algorithm balances by monitoring the source status of each server and analyzing the load capacity adjustment of each node.

Through the above analysis and comparison of several load balancing algorithms, this article chooses a dynamic load balancing algorithm to achieve resource load balancing. The collection of PM (physical machine) and VM (virtual machine) data of each node in the cluster is the basis of load balancing, because algorithm balancing can be completed through the loading function of each node, and finally load balancing is determined. Because load balancing is implemented dynamically, real-time collection is required when collecting node resource information. Through analysis of the collected data, the causes of uneven load of virtual machine resources can be efficiently analyzed and processed. While collecting nodes, it is necessary to monitor the resource status of each node in real time, and the related scheduling work can be realized at the end through monitoring.

## 3. Ant Colony Algorithm

For the network, load balancing technology is the basis for the stable operation of the network and the saving of operating resources. The article will use ant colony algorithm to achieve load balancing of network links. At the same time, through the experimental analysis and selection of some parameters in the ant colony algorithm, we finally obtain a better load balancing effect.

The principle of the ant colony algorithm is that when insects carry food, they will leave a recognizable pheromone on the street, and other ant colonies can recognize this pheromone and know the concentration of the pheromone. Then, a pathway with a high pheromone concentration will be more likely to be selected, other ant colonies will pay attention to this pathway accordingly, and the pheromone concentration will increase accordingly, thus forming a positive feedback system. Therefore, the pheromone on the street will also change over time, and the pheromone concentration will decrease accordingly, which will affect the choices of other insects. Then, in the area where the insects search for food and bring the food back to the nest, because a large number of ants continue to carry the food, it is likely that the shortest route from the nest to the foraging location will appear, and the food will eventually be collected successfully [15].

The specific expression of the ACO algorithm is shown in the following equation:

(1) $$\begin{array}{c} P_{ij}^{K}\left(t\right)=\left\{\begin{array}{c} \tau_{ij}^{\alpha }\left(t\right)*\kappa_{ij}^{\beta }\left(t\right)\\ s\in \text{allowedk }\tau_{is}^{\alpha }\left(t\right)*\kappa_{is}^{\beta }\left(t\right),s\in \text{allowedk}.\\ 0,s\in \text{allowedk} \end{array}\right) \end{array}$$

Among them, *κ*_*ij*_^*β*^ is the heuristic factor of the distance perceived by the ants between *i* and *j*, and the size is related to the distance between the two cities.

(2) $$\begin{array}{c} \kappa_{ij}\left(t\right){=}_{d_{ij}}^{1}. \end{array}$$

It can be seen from this formula that if the distance between (*i*, *j*) is smaller and the heuristic factor is greater, then the transition probability is greater. The calculation formula of *d*_*ij*_ is as follows:

(3) d=ijxi−xj2+yi−yj2.

At all times in the ACO algorithm, there are pheromone updates on the path. With the following equation, the pheromones are updated:

(4) $$\begin{array}{c} \tau_{ij}\left(t+1\right)=\left(1-\gamma \right)*\tau_{ij}\left(t\right)+\gamma *\Delta \tau_{ij}\left(t,t+1\right). \end{array}$$

*γ* represents the pheromone volatilization coefficient between (0–1). The specific formula of is as follows:

(5) $$\begin{array}{c} \Delta \tau_{ij}\left(t,t+1\right)=\sum_{k=1}^{m}\Delta \tau_{ij}\left(t,t+1\right). \end{array}$$

Accordingly, in order to prevent the ants from traversing town *i* again after traversing town *i*, a contraposition table would be added to the ant colony algorithm to record the towns that have been traversed by the ant in a time period. After the round of traversal is complete, it will be cleared and a new round of traversal will be performed. The calculation model formula is as follows:

(6) $$\begin{array}{c} \Delta \tau_{ij}\left(t,t+T\right)=\left\{\begin{array}{c} K,\\ Ln,\\ 0, \end{array}\right)\begin{array}{c} k\in \left(i,j\right),\\ \text{other}. \end{array} \end{array}$$

In the initial stage of path search, ants can choose more paths to ensure the diversity of solutions and expand the search space of solutions. Here, the *k*-th ant can transition from state *i* to state *j* with the following probability:

(7) $$\begin{array}{c} j=\left\{\begin{array}{c} \begin{array}{cc} \arg & \max\left\{\tau {\left(\gamma \right)}^{\rho }\right\}, \end{array}\\ J. \end{array}\right) \end{array}$$

The article studies the mathematical principles, theories, and related applications of the ant colony algorithm. In particular, it proposes an improved ant colony algorithm for the shortcomings of the algorithm that is prone to stagnation, and finally verifies its effectiveness with specific TSPs.

Through simulation experiments, the influence of parameter range on the optimal solution is studied. The main parameters are as follows: *α* is the relative importance of pheromone (pheromone heuristic factor); *β* is the relative importance of heuristic factor (expected heuristic factor); *ρ* is the pheromone volatilization coefficient ((1− *ρ*) represents the persistence coefficient of pheromone); *m* is the number of ant colonies.

In the cloud computing environment, the problem of resource allocation is still a combination optimization problem. In the cloud computing environment, there are many factors affecting resource allocation, which correspond to the length of the intercity path in the traveling salesman problem. From the above application experiment of genetic ant colony algorithm (GACA) which improves ant colony algorithm through genetic algorithm, it is known that the fusion of intelligent algorithms is a more efficient and correct way to solve the problem. However, the merged algorithm can still have premature convergence in the later stage. Therefore, we need to maintain the diversity of the population in the iterative process and expand the search solution space to a certain extent, so as to prevent the occurrence of premature convergence to a certain extent. The definition of matching factor is introduced to express the matching degree of each task and each resource node.

(8) $$\begin{array}{c} {\text{Match}}_{ij}=\frac{1}{\sqrt{\sum_{n=1}^{4}{\left(T_{xi}-V_{yj}\right)}^{2}}}. \end{array}$$

Supposing *X* is a mapping sequence of tasks and resources, the degree of load balance is defined as follows:

(9) $$\begin{array}{c} \text{Load}\left(X\right)=\sqrt{\sum_{i=1}^{n}{\left(1-C_{1}\frac{Y_{i}}{Lv_{i}}\right)}^{2}}. \end{array}$$

Among them, *Y*_*i*_ indicates how many tasks are allocated to resource node *i*.

Approximate nondeterministic tree search (ANTS) is an ACO algorithm that uses mathematical programming ideas. The ANTS algorithm uses a new action selection rule and pheromone update rule, as shown in the following formula:

(10) $$\begin{array}{c} p_{ij}^{k}=\frac{\gamma \tau_{ij}+\left(1-\gamma \right)\eta_{ij}}{\sum_{i\in N_{i}^{k}}\gamma \tau_{ij}+\left(1+\gamma \right)\eta_{ij}},\\ \tau_{ij}\leftarrow \tau_{ij}+\underset{k=1}{\sum }\Delta \tau_{ij}^{k},\\ \Delta \tau_{ij}^{k}=\left\{\begin{array}{c} \theta \left(1-\frac{C^{k}-LB}{L_{\text{avg}}-LB}\right)\\ 0 \end{array}\right). \end{array}$$

Among them, *θ* is a parameter, and LB is an optimal solution calculated at the beginning of the algorithm.

For any given data, there is a uniquely determined membership function value *μA*(x) ∈ [0,1] corresponding to it, which can be expressed as follows:

(11) $$\begin{array}{c} \mu \tilde{A}\left(x\right):X⟶\left[0,1\right]. \end{array}$$

Usually, the expression is as follows:

(12) $$\begin{array}{c} \tilde{A}=\frac{\mu_{\tilde{A}}\left(x_{1}\right)}{x_{1}}+\frac{\mu_{\tilde{A}}\left(x_{2}\right)}{x_{2}}+\cdots +\frac{\mu_{\tilde{A}}\left(x_{n}\right)}{x_{n}}. \end{array}$$

This kind of representation can be represented by sequential even representation:

(13) $$\begin{array}{c} \tilde{A}=\left\{\left(x_{1},\mu_{\tilde{A}}\left(x_{1}\right)\right),\left(x_{2},\mu_{\tilde{A}}\left(x_{2}\right)\right),\ldots ,\left(x_{n},\mu_{\tilde{A}}\left(x_{n}\right)\right)\right\}\text{,} \end{array}$$

or using vector notation:

(14) $$\begin{array}{c} \tilde{A}=\left\{\mu_{\tilde{A}}\left(x_{1}\right),\mu_{\tilde{A}},\ldots \mu_{\tilde{A}}\left(x_{n}\right)\right\}. \end{array}$$

In the cloud computing system *t*, there are *N* tasks that need to be allocated to *M* nodes for processing, and the current load status of each server is different. The load balancing strategy is to find the most reasonable task allocation plan, so that the average processing time of tasks is the shortest, and the service quality of the cloud computing system is improved. The load deviation rate is used to measure the system load distribution after assigning tasks, and the load deviation rate is calculated as follows:

(15) $$\begin{array}{c} E\left(x1,x2,\ldots ,xn\right)=\frac{1}{n}\sqrt{\sum_{i=1}^{M}e_{i}^{2}}. \end{array}$$

Among them, *M* represents the predicted value of the resource load required on the *i*-th server under this task allocation plan, and the calculation formula is as follows:

(16) $$\begin{array}{c} e_{i}=f_{i}\left(x_{i},L_{i}\right)-F\left(x_{1},x_{2},\ldots ,x_{n}\right). \end{array}$$

Among them, *f*_*i*_(*x*_*i*_, *L*_*i*_) represents the predicted value of resource load required on the *i*-th server under this task allocation plan, and the calculation formula is as follows:

(17) $$\begin{array}{c} f_{i}\left(x_{i},L_{i}\right)=\left(x_{i}+1\right)*L_{i}. \end{array}$$

In the current server running state, the calculation formula for the impact of allocating a unit of computing resource on the load is as follows:

(18) $$\begin{array}{c} F\left(x_{1},x_{2},\ldots ,x_{n}\right)=\frac{1}{M}\sum_{i=1}^{M}f_{i}\left(x_{i},L_{i}\right). \end{array}$$

According to the above calculation formula, the load deviation rate takes a value in the range of 0 to 1. The smaller the value, the more balanced the load distribution of the cloud computing system, and the better the performance of the current system [16].

## 4. Experiments and Results of Cloud Computing Load Balancing

### 4.1. Experiment Preparation

The cloud computing simulation platform is selected to conduct experimental analysis and evaluation of the cloud computing load balancing process based on virtual machine relocation. The main performance indicators are the load balance of CPU, memory, and other sources and the average operating time. By monitoring the load situation in the network in real time, the ant colony algorithm can give the forwarding link with the smallest load, so as to realize the relative balance of dynamic link load. This can optimize the configuration of limited network resources and effectively solve the problems of low network bandwidth utilization and low throughput. In order to simplify the processing and reflect the reliability of the experimental results of different strategies, in this simulation experiment, the cloud computing data center is configured with the same type of servers, virtual machines with the same parameters, and the same network environment and performs a set of the same tasks. The specific conditions are shown in Table 1.

It is measured by the load standard deviation for the CPU and memory of the system. Their corresponding utilization standard difference will be calculated by detecting the CPU or memory utilization at a given time for each host.

The level of memory load balancing is compared between layered management-based virtual machine migration strategy (MLVM) and agent-based virtual machine migration strategy (PAVM). After that, the entire CPU utilization of the system is read at different time points, and the standard deviation of the system CPU load balance is calculated. The experimental results are shown in Table 2.

Through experiments, the task response time for different task requests is counted, and the average task response time is calculated. The average task response time of the two strategies is shown in Table 3.

### 4.2. Algorithm Optimal Solution

We perform statistics on the optimal solutions for different *α* values in the ant colony algorithm, and the results are shown in Figure 5.

The heuristic factor *α* characterizes the relative importance of the pheromone accumulated by the ants in the process of constructing the solution for the path selection in the ant search. The larger the value of *α*, the more likely the ants will pick the previous paths they traveled and the searching paths will be less stochastic. When *α* takes different values, the corresponding optimal iterative optimal solution and number of iterations are shown in Figure 6. When *α* = 1, the iterative optimal solution gets the minimum value, and then as *α* increases, the iterative optimal solution value also increases; the number of iterations also decreases as *α* increases. This reflects the overall impact of *α* on the algorithm, that is to say, the larger the value of *α*, With the greater likelihood of selecting previously traveled paths, the more likely the ants are to choose previously walked paths; there will be less randomness in the search paths, they will converge faster, and they will be easily restricted to limiting themselves to locally optimal solutions.

We carry out statistical analysis on the load quantity of each resource of MLVM and PAVM, and the results are shown in Figure 7.

It can be seen that PAVM accepts the criteria to increase the possibility of finding a better allocation method, which is subject to certain restrictions on the execution time of the algorithm, but there is a certain improvement in the scheduling time. We compare the task time spans of several most commonly used algorithms, such as ant colony algorithm, genetic ant colony algorithm, and improved algorithm, and the results are shown in Figure 8.

In a load balancing system, validity is an important criterion for judging the quality of its algorithm, so it is particularly important to verify this criterion. Due to the instability of the experimental results, the method of seeking a tie for each set of experiments is used to obtain the final result. We judged the effectiveness of different methods by the response time when reading files of different sizes. The experimental results are shown in Figure 9.

It can be seen that the response time for reading each file varies, and this time is not completely related to the file size, which means that not all large files have a long response time, and not all small files have a short response time. However, in the ACO algorithm, the average response time is about 30% lower than that in other algorithms. This shows that the ACO algorithm can play a role.

## 5. Discussion

In order to avoid data loss and improve system reliability, copy technology is usually used in cloud storage systems. The copy technology is to make multiple copies of a data block, store them on multiple nodes, and use data redundancy to ensure data reliability. The use of copy technology can well solve the load balancing problem of the system. Multiple copies are distributed on different server nodes. By accessing the copy, the load of a single server node is distributed to multiple nodes, thereby reducing the load of the nodes and achieving load balancing.

The ant colony optimization algorithm has undergone more than ten years of development since it was proposed and has achieved remarkable results in algorithm theory research and application. Its application scope involves various optimization fields such as routing problems, allocation problems, scheduling problems, subset problems, machine learning problems, and emergence of ant colony algorithm bionic hardware, showing the strong vitality and broad development of ant colony optimization algorithm prospect.

With the continuous update and development of computer technology, the number of users has doubled, the architecture of traditional IP networks has become more and more complex, and the development of the network structure is relatively lagging. In this paper, the load balance is realized by using the ant colony algorithm, which is implanted in the controller, and the network load is monitored in real time through the traffic monitoring software. Through the execution of the ant colony algorithm in the controller, the data stream will be transmitted along the link with the least load at a certain moment, which can effectively use network resources, reduce network congestion, increase network throughput, and realize network dynamic load balancing of each link in the network. We also carried out theoretical experimental research and analysis on the heuristic factor, the pheromone volatilization coefficient, and the number of ants in the ant colony algorithm. Through the selection of parameters, the performance of the ant colony algorithm was improved, and the load balancing was also able to obtain better results. We conduct load balancing experiments on the self-defined network topology. Through the analysis of experimental data, the introduction of ant colony algorithm can achieve dynamic load balancing of each link.

## 6. Conclusion

For the purpose of this paper, we will be looking at the allocation of resources for cloud computing. According to the existing algorithm, the intelligent algorithm is fused, and the pheromone initial allocation of the ant colony algorithm is introduced to solve the blind search problem and avoid the later local optimal solution problem. The improved algorithm was applied to the specific problem of cloud computing resource allocation, and experimental calculation and analysis were performed. It was found that the time span performance and resource load degree had relatively good results, which proved the applicability of the algorithm. The improved algorithm proposed in this paper has certain performance optimization but also has certain disadvantages. The algorithm becomes slightly more complicated and has a great test on the execution speed. Moreover, the actual situation should be fully considered in the actual application process; for example, issues such as more diverse and dynamic user needs and complexity of resources require comprehensive consideration of the needs and interests of users and providers. In addition, the ant colony algorithm is often aimed at a certain type of special problem, and its versatility is poor. In future research, if we want to use the ant colony algorithm in other fields, we need to improve its universality. In addition, the research in this paper only considers the small network with few hosts and single controller and does not consider the load balancing of the large network with multiple hosts and multiple controllers, and the researcher hopes that this part of the research can be completed through corresponding experiments in the future.

## Figures and Tables

**Figure 1:** Cloud computing system.

**Figure 2:** Cloud computing hierarchy.

**Figure 3:** Cloud storage system structure.

**Figure 4:** Load balancing architecture.

**Figure 5:** The value of the heuristic factor solution.

**Figure 6:** The relationship between the optimal solution and the number of iterations.

**Figure 7:** The amount of load for each resource.

**Figure 8:** Task time span.

**Figure 9:** Response time for different file sizes.

**Table 1:** Comparative experimental parameters.

Parametric variable	Parameter value
Host quantity	40
Host core number	2
Host memory	4 GB
Core computing speed	2 GHz
Initial number of virtual machines	250
Number of tasks	300
Total CPU demand	2500 GHz
Total memory requirements	4 GB

**Table 2:** System CPU load standard deviation at different time points.

Time/s	MLVM CPU load standard deviation	PAVM CPU load standard deviation
100	0.23	0.24
200	0.20	2.25
300	0.23	0.24
400	0.21	0.23
500	0.18	0.21
600	0.16	0.21
700	0.10	0.15
800	0.09	0.14

**Table 3:** Task response time.

Number of tasks	MLVM average response time	PAVM average response time
20	5.97	5.99
50	6.01	6.02
100	6.23	6.21
150	6.51	6.65
200	7.34	7.82
250	7.64	7.92
300	8.01	9.25
400	8.54	9.73

## Data Availability

The data used to support the findings of this study are available from the author upon request.
